RETRACTED

# Circular RNA circCCDC66 Contributes to Malignant Phenotype of Osteosarcoma by Sponging miR-338-3p to Upregulate the Expression of PTP1B

**DOI:** 10.1155/2020/4637109

**Published:** 2020-08-10

**Authors:** Deng Xiang, Yugang Li, Yanshui Lin

**Affiliations:** Department of Orthopaedics, The First Affiliated Hospital of Chengdu Medical College, Chengdu, Sichuan 610500, China

## Abstract

In recent years, the mechanism of cancer research has become hotspots of life science and medicine, especially due to the rapid development of molecular medicine and bioinformatics research. Similarly, the molecular mechanism also has received increasing attention in osteosarcoma (OS) research. Also, a considerable amount of research confirmed that circular RNAs (circRNAs) could regulate cancer cell growth and metastasis. This study aimed to explore the effect of a circRNA, circCCDC66, on OS and reveal its potential molecular mechanism. High circCCDC66 expression level was found in OS patient-derived tissue samples and OS cell lines by qRT-PCR. The abilities cell proliferation and metastatic of U2OS and SW1353 cells were then assessed by Cell Counting Kit-8 and transwell assay, respectively. The interaction between circCCDC66 and its target miRNAs were verified by the dual-luciferase reporter assay. Through functional experiments, we found that circCCDC66 knockdown promoted the inhibition of cell proliferation and metastatic of OS cell lines. From mechanistic perspective, circCCDC66 upregulated PTP1B by sponging miR-338-3p. Collectively, our findings demonstrated that circCCDC66 contributed to malignant behaviors of OS cells by miR-338-3p/PTP1B pathway, which suggested circCCDC66/miR-338-3p/PTP1B axis might be a potential therapeutic target.

## 1. Background

In addition to the mRNA involved in coding, there are also a large number of noncoding RNAs. A class of RNAs with circular structures that are very different from other noncoding RNAs are called circRNAs [1]. circRNA was discovered as early as about 40 years ago by electron microscopy [2]. Limited by the technical means at that time, further studies could not be conducted. However, recent advances in molecular biology, particularly in sequencing and nucleic acid synthesis and splicing, have created opportunities for circRNA research. Although many questions about circRNA have not been answered, scholars have gradually gained new understanding of circRNA [3]. As for the origin of circRNA, with the deepening of research, we gradually realize the particularity and complexity of its biogenesis mechanism. circRNAs can be formed by linear RNA splicing, direct back-splicing pathway, and lariat driven pathway [4]. Similarly, compared with previous studies, researchers have also made some progress in the study of circRNA functions [1, 5]. circRNA can combine the competition of miRNA with the downstream target genes to achieve the inhibitory effect of miRNA, thus modulating the downstream target genes expression [6]. For example, circRNA ciRS-7 has a spongy effect on miR-7, strongly inhibiting miR-7 activity, which then leads to increased miR-7 target expression levels [7]. In addition, intron circRNAs can affect parental genes transcription in the nucleus. circRNA can isolate or regulate protein functions by interacting with proteins. The exon circRNA itself is a product of the regulatory mechanism, and it is spliced into a ring, so the expression of its parent genes must be affected [5]. Of course, circRNA must also have other features that we have not yet learned in detail.

RETRACTED

Numerous studies have shown that the expression levels of certain circRNAs vary from cancer to normal tissues. These results are important because they provide important avenues for studying the mechanisms of cancer progression and expression, as well as new potential approaches for screening, diagnosing, monitoring, and treating cancer [8, 9]. For example, in gastric cancer tissues, hsa_circ_0003159 is significantly downregulated, which is negatively regulated by the development of cancer, such as distant metastasis of tumor tissues, thus serving as a potential tumor biomarker for GC patients [10]. In bladder cancer tissues and cell lines, the expression of circSLC8A1 is downregulated and is related to the pathological stage and histological grade of bladder cancer. circSLC8A1 can directly interact with miR-130b/miR-494, regulate the expression of PTEN, and inhibit the progression of bladder cancer [11]. Meanwhile, significant upregulation of circRNA-000284 was found in cervical cancer cells, which were positively correlated with the proliferation and metastasis capacity of cancer cells and also affected the cell cycle process of cancer cells [9]. In addition, in bladder cancer, the forced expression of circRNA BCRC4 was found to enhance the expression level of miR-101 and inhibit the expression of the downstream gene EZH2, thus playing the role of tumor suppressor [8]. The results offer new potential strategies for the treatment of bladder cancer.

The important factor of tumorigenesis is that the cells get rid of normal regulation and have the potential to resist apoptosis and unlimited proliferation [12]. Osteosarcomas are no exception [13]. Although osteosarcomas have less incidence rate than other common cancers, they often occur in children and adolescents and are more aggressive [14]. Osteosarcoma is also characterized by strong invasiveness and strong resistance to chemotherapy, resulting in a poor prognosis and a high recurrence rate [15]. These characteristics cause much trouble to orthopedic doctors and also make the patient's quality of life low and later life unsatisfying [16]. This situation calls for new markers and methods.

RETRACTED

Differential expressions of circCCDC66 in osteosarcoma and normal tissues were analyzed to explore the role of circCCDC66 in osteosarcoma cells. The present study also assayed a series of in vitro experiments. In this study, si-circCCDC66 was transfected into osteosarcoma cells SW1353 and U2OS, and the expression of circCCDC66 was silenced to investigate the roles of circCCDC66 in cell growth and metastasis. In addition, the mechanism of circCCDC66 was investigated by bioinformatics analysis and luciferase reporter assay. We expected this study to provide more potential methods for the detection, diagnosis, and monitoring of osteosarcoma.

## 2. Material and Method

### 2.1. Patients and Tissue Samples

Totally, 12 OS patients undergoing complete resection surgery in our hospital between 2016 and 2020 were included in present project, which was agreed upon by the Ethics Committee of our Hospital. All tissue samples used in this study were administered with the written informed consent of the OS patients.

### 2.2. OS Cell Culture and Transfection

SW1353 and U2OS were cultured in RPMI-1640 supplemented with 10% FBS (BI, Israel) and 1% penicillin/streptomycin (Sigma-Aldrich) at 37°C under 5% CO_2_ atmosphere. The transfection was conducted using Lipofectamine2000 kit according to the product instructions.

### 2.3. Cell Counting Kit-8 (CCK-8) Assay

SW1353 and U2OS cells transfected with indicated mimics were seeded into 96-well plates. Then, CCK-8 (Dojindo Chemical Laboratory, Kumamoto, Japan) was added to a 96-well plate at 10 *μ*L per well and its absorbance was measured at 450 nm according to the instruction manual [17].

### 2.4. Cell Invasion and Cell Migration

Cell invasion was detected using a 24-well transwell chamber (Corning, New York, USA) with coated with Matrigel (BD Biosciences). Cell migration was detected using a 24-well transwell chamber (Corning, New York, USA). Briefly, SW1353 and U2OS cells transfected with indicated mimics in 100 *μ*L serum-free medium were plated in the top chamber. Next, 600 *μ*L complete medium was added to the lower chambers. 48 h later, the invaded and migrated cells were counted according to the manufacturer's instructions [18].

### 2.5. qRT-PCR Assay

qRT-PCR assay was applied to detect the differential expression of candidate genes with the SYBR Green PCR kit, following the RNA extraction with TRIzol, and reverse transcription with Primer Script RT mix. All regents were purchased from Takara Company according to the instruction manual. GAPDH was used as an internal control and relative gene expression was determined with the 2^−ΔΔCt^ method.

RETRACTED

### 2.6. Dual-Luciferase Reporter Assay

The WT or MUT circCCDC66 or PTP1B-3′UTR containing a miR-338-3p binding sequence was cloned into the pmirGLO Vector (Promega, WI, USA). Then, the construct vectors were transfected into 293 T cells with control or miR-338-3p mimics. Subsequently, luciferase activity was detected with a dual-luciferase reporter assay kit (Promega) according to the manufacturer's instructions.

### 2.7. Bioinformatics Analysis

RegRNA 2.0 (http://regrna2.mbc.nctu.edu.tw) was used as a widely used regulatory RNA motifs identification tool for bioinformatics analysis. The predictive results were presented via a graphical interface.

### 2.8. Statistical Analysis

All statistical analyses were analyzed using GraphPad Prism 7.0 software (GraphPad Inc., USA). Statistics were analyzed by the Student's *t* test with a value of significance set at *p* < 0.05.

## 3. Results

### 3.1. circCCDC66 Expression Was Increased in OS Tissues and Cells

In order to evaluate whether circCCDC66 was a circRNA, we detected circCCDC66 and CCDC66 mRNA expression after RNase R digestion. As presented in Figure 1, we found circCCDC66 was resistant to RNase R digestion compared with the linear form. Subsequently, the expression level of circCCDC66 was analyzed through qRT-PCR assay in OS tissues and cell lines to understand the potential roles of circCCDC66 in OS. Results showed that circCCDC66 levels were higher in the OS tissues than those in the normal tissues (Figure 1(c)). Moreover, similar results also appeared in cell lines, with the expression of circCCDC66 being much more abundant in OS cells SW1353 and U2OS than in normal cells hFOB1.19 (Figure 1(d)). These results suggested that circCCDC66 might be related to OS.

### 3.2. Bioinformatics Analysis of circCCDC66 in OS

Furthermore, we predicted the potential functions of circCCDC66 in OS using ceRNA and bioinformatics analysis. As shown in Figure 2, the top biological processes related to circCCDC66 included chromosome organization and biogenesis, regulation of endocytosis, transport, regulation of immune response, organogenesis, regulation of translation, vesicle-mediated transport, and regulation of gene expression and epigenetic. The top KEGG pathways included signaling by EGFR, signaling by NGF, signaling by robo receptor, cell cycle, mitotic, PI-3K cascade, downstream signaling of activated FGFR, signaling by insulin receptor, and DNA replication.

RETRACTED

### 3.3. circCCDC66 Promoted OS Cell Proliferation, Migration, and Metastasis

Next, we designed siRNA oligonucleotides targeting the unique back splice junction to knockdown circCCDC66 expression in OS. The expression of circCCDC66 was successfully knockdown using si-circCCDC66. The specific knockdown contributed to a remarkably reduction of cell proliferation rate in SW1353 and U2OS using CCK-8 assay (Figures 3(a) and 3(b)). In addition to cell proliferation, transwell assay results demonstrated that the silencing of circCCDC66 significantly reduced cell abilities of migration and invasion. As presented in Figure 3, the migrated and invaded cells numbers were suppressed in circCCDC66 knockdown group compared to the control group.

### 3.4. circCCDC66 Increased PTP1B Expression by Sponging and Inhibiting miR-338-3p in OS

Cytoplasmic circRNAs enhanced targets expression by acting as ceRNAs to sponge miRNAs. Subcellular fractions qRT-PCR analysis indicated that circCCDC66 was more distributed in the cytoplasm (Figure 4(a)). Bioinformatics analysis predicted that hsa-miR-141-3p, hsa-miR-185-5p, hsa-miR-200a-3p, and miR-338-3p might have interacted with circCCDC66 using online miRNA binding databases (Figures 4(b)– 4(d)). The dual-luciferase reporter assay showed that miR-338-3p significantly reduced luciferase activity of both SW1353 and U2OS cells overexpressing circCCDC66-WT plasmids, but not circCCDC66-MUT plasmids (Figure 4(e)).

The further validation of the interaction between miR-338-3p and circCCDC66 indicated miR-338-3p levels were remarkably induced by circCCDC66 knockdown in both SW1353 and U2OS cells (Figure 4(f)).

Then, we explored the molecular function of miR-338-3p in OS. The overexpression of miR-338-3p contributed to a remarkable reduction of cell proliferation rate in SW1353 and U2OS using CCK-8 assay (Figures 5(a) and 5(b)). In addition to cell proliferation, transwell assay results demonstrated that overexpression of miR-338-3p appreciably reduced cell abilities of migration and invasion (Figure 5(c)).

Then, the prediction showed that miR-338-3p could directly bind to PTP1B. Overexpression or knockdown of miR-338-3p significantly suppressed or enhanced PTP1B expression in SW1353 cells (Figure 6(a)). Dual-luciferase reporter assay showed that miR-338-3p overexpression remarkably decreased the luciferase activity of both SW1353 and U2OS cells transfected by PTP1B-WT instead of PTP1B-MUT (Figure 6(b)). Moreover, the knockdown of circCCDC66 or the upregulation of miR-338-3p could inhibit the expression and luciferase activity of PTP1B (Figures 6(c) and 6(d)). These findings demonstrated that circCCDC66 increased PTP1B expression by sponging and inhibiting miR-338-3p in OS.

RETRACTED

## 4. Discussion

Clinical markers played important roles in cancer diagnosis and disease progression monitoring [19]. The common broad-spectrum tumor markers of proteins include oncoembryonic antigen and alpha-fetoprotein [20]. Similarly, studies have demonstrated the potential value of Aurora A kinase as a tumor marker due to its high expression in OS and the potential of plasma 4 integrin and ezrin as tumor markers in the initial stage of OS development [21–23]. Recently, with the rapid development of biology, more and more RNA biomolecules are used as clinical markers of cancer [24]. For example, microRNA-195, microRNA-223, microRNA-221, microRNA-421, and microRNA-203 in serum are differently expressed in OS tissues, indicating that they can be used as a new biomarker for screening OS to predict poor prognosis and monitor the progress of cancer [17, 25–28]. In the present study, we found that circCCDC66 was overexpressed in tumor cells compared to normal tissues. After silencing, the growth and metastasis of tumor cells were significantly inhibited. Therefore, circCCDC66 was positively correlated with the occurrence, development, and metastasis of OS and had potential application value as a marker for screening and monitoring OS.

Previous studies show that circCCDC66 also plays a role in colon cancer [29]. circCCDC66 expression in colon cancer is higher than in normal tissue and related to poor prognosis. Further studies have indicated that circCCDC66 contains multiple different binding sites of miRNA, and the overexpression of circCCDC66 acts as a miRNA sponge to interfere with miRNA-33b and miR-93, inhibiting its binding to downstream target genes, leading to high expression of downstream target genes, thereby increasing the level of MYC protein and promoting the proliferation, invasion, and metastasis of colon cancer [30]. Another study also showed that in radiation-resistant colon cancer tissues, circCCDC66 was significantly upregulated and miR-338-3p was significantly downregulated, so circCCDC66 could negatively regulate miR-338-3p to promote radiation resistance in colon cancer tissues [6].

miRNAs, one of the abundant noncoding RNAs in cells, are a class of microRNAs encoded by less than 30 nucleotides [31]. The main mechanism of miRNA is the incomplete binding with the 3′-UTR of the downstream mRNA, thus inhibiting the gene expression of the latter, namely protein synthesis [32]. miRNA-mediated regulation of gene expression is complex, which can compete with mRNA for RNA-binding proteins to inhibit translation, and such inhibition is sometimes affected by the selective binding mechanism of RNA-binding proteins, resulting in poor effect. In some cases, miRNA involved in regulation will be stimulated and lead to self-degradation, which will lead to the reactivation of inhibited mRNA [33]. The miR-338-3p has also been found to play an important role in numerous cancers. For example, miR-338-3p suppressed the growth of neuroblastoma by modulating the downstream gene PREX2a, regulated the occurrence and development of gastric cancer cells by participating in ZEB2, MACC1/Met/Akt and SSX2IP regulatory pathway [34, 35]. Similarly, in this study, we found through knockout experiments that the downregulation of circCCDC66 expression enhanced the interaction between miR-338-3p and PTP1B and inhibited the proliferation and metastasis of OS cells.

RETRACTED

Our reports revealed the functions and mechanism of circCCDC66 in the development of OS. As one of the malignant tumors, OS urgently needs further research to find more screening, diagnosis, and treatment methods, so as to improve the survival time and quality of life of patients. Our study explored the role of circRNA in OS, providing potential strategies for the screening and treatment of OS. However, more studies are needed to explore the more detailed regulatory processes in the development of OS.

## Figures and Tables

**Figure 1:** circCCDC66 expression was increased in OS tissues and cells. (a) qRT-PCR assay of circCCDC66 after treatment with RNase R. (b) qRT-PCR assay of CCDC66 mRNA in OS cells treated with RNase R. (c) The relative expression levels of circCCDC66 in 12 pairs of OS tissues and matched noncancerous tissues by qRT-PCR assay. (d) Detection of circCCDC66 expression levels in OS cell lines by qRT-PCR assay. ∗*p* < 0.05, ∗∗*p* < 0.01, ∗∗∗*p* < 0.001.

**Figure 2:** Bioinformatics analysis of circCCDC66 in OS. (a) The top biological processes related to circCCDC66. (b) The top KEGG pathways.

**Figure 3:** circCCDC66 promoted OS cell proliferation, migration, and metastasis. (a, b) Effect of CCDC66 knockdown on cell proliferation. (c–f) Comparison of OS cells transfected with the si-circCCDC66 and the control group in transwell assay. ∗*p* < 0.05, ∗∗*p* < 0.01.

**Figure 4:** circCCDC66 acted as a sponge for miR-338-3p. (a) circCCDC66 was more distributed in the cytoplasm. (b, c) The relative expression levels of 4 miRNAs in the circCCDC66 probe group and the control probe group in SW1353 and U2OS cells, respectively. (d) Predicted binding sites for miR-338-3p with the circCCDC66 and the design of wild-type (WT) and mutant (MUT) circCCDC66 luciferase reporter vector constructs. (e) Effect of miR-338-3p mimics on circCCDC66 WT and circCCDC66 MUT was detected through dual-luciferase reporter assay. (f) The expression levels of miR-338-3p in SW1353 and U2OS cells transfected with the si-circCCDC66 or si-NC was detected by qRT-qPCR assay. ∗∗*p* < 0.01.

RETRACTED

**Figure 5:** Effects of miR-338-3p on cellular physiological functions. (a, b) Cell proliferation was determined in SW1353 and U2OS cells transfection with miR-338-3p by CCK-8 assays. (c) Comparison of the cell metastatic capability in SW1353 and U2OS cells transfected with the miR-338-3p mimic or miR-NC by transwell assay. ∗*p* < 0.05, ∗∗*p* < 0.01.

**Figure 6:** circCCDC66 increased PTP1B expression by sponging and inhibiting miR-338-3p in OS. (a) Knockdown of miR-338-3p significantly enhanced PTP1B expression in OS cells. (b) miR-338-3p overexpression decreased the luciferase activity of both SW1353 and U2OS cells transfected by PTP1B-WT. (c) Knockdown of circCCDC66 or the upregulation of miR-338-3p can inhibit the expression of PTP1B mRNA. (d) Relative luciferase activities of 293 T cells cotransfected with PTP1B 3′-UTR-MUT, PTP1B 3′-UTR-WT and Mock, si-circCCDC66, miR-NC, or miR-338-3P vector were analyzed through luciferase reporter experiments. ∗*p* < 0.05, ∗∗*p* < 0.01.

## Data Availability

All the related data could be provided if any qualified authors required.
